# Ultrasonic Image Features under the Intelligent Algorithm in the Diagnosis of Severe Sepsis Complicated with Renal Injury

This article has been retracted.

**DOI:** 10.1155/2022/2310014

**Published:** 2022-08-11

**Authors:** Leiming Xu, Xin Wang, Pu Pu, Suhui Li, Yongzheng Shao, Yong Li

**Affiliations:** ^1^Department of Emergency Medicine, Binhai County People's Hospital, Binhai, 224500 Jiangsu, China; ^2^Department of Intensive Care Unit, Binhai County People's Hospital, Binhai, 224500 Jiangsu, China

## Abstract

This research was aimed at analyzing the diagnosis of severe sepsis complicated with acute kidney injury (AKI) by ultrasonic image information based on the artificial intelligence pulse-coupled neural network (PCNN) algorithm and at improving the diagnostic accuracy and efficiency of clinical severe sepsis complicated with AKI. In this research, 50 patients with sepsis complicated with AKI were collected as the observation group and 50 patients with sepsis as the control group. All patients underwent ultrasound examination. The clinical data of the two groups were collected, and the scores of acute physiology and chronic health assessment (APACHE II) and sequential organ failure assessment (SOFA) were compared. The ultrasonic image information enhancement algorithm based on artificial intelligence PCNN is constructed and simulated and is compared with the maximum between-class variance (OSTU) algorithm and the maximum entropy algorithm. The results showed that the PCNN algorithm was superior to the OSTU algorithm and maximum entropy algorithm in the segmentation results of severe sepsis combined with AKI in terms of regional consistency (UM), regional contrast (CM), and shape measure (SM). The acute physiology and chronic health evaluation (APACHE II) and sequential organ failure assessment (SOFA) scores in the observation group were substantially higher than those in the control group (*P* < 0.05). The interlobular artery resistance index (RI) in the observation group was substantially higher than that in the control group (*P* < 0.05). Moreover, the mean transit time (mTT) in the observation group was significantly higher than that in the control group (4.85 ± 1.27 vs. 3.42 ± 1.04), and the perfusion index (PI) was significantly lower than that in the control group (134.46 ± 17.29 vs. 168.37 ± 19.28), with statistical significance (*P* < 0.05). In summary, it can substantially increase ultrasonic image information based on the artificial intelligence PCNN algorithm. The RI, mTT, and PI of the renal interlobular artery level in ultrasound images can be used as indexes for the diagnosis of severe sepsis complicated with AKI.

## 1. Introduction

Acute kidney injury (AKI) refers to a clinical syndrome in which a sudden decrease in the glomerular filtration rate leads to the accumulation of nitrogenic products in a short period of time due to various reasons, resulting in the disturbance of water, electrolyte, and acid-base balance and the rapid development of systemic complications [1–3]. Severe sepsis and septic shock are the main causes of AKI in China, and the detection rate of AKI is related to sepsis. A multicenter prospective cohort study involving 1,255 patients with severe sepsis showed that the prevalence of AKI was 31.6%, among which severe sepsis and septic shock accounted for 44.9%, and the 90-day fatality rate was 41.9% [4, 5]. Panuccio et al. [6] conducted a prospective observational study on 10 severe sepsis patients and found that 30.6% (116/379) of them had sepsis-related AKI. Obviously, the incidence of AKI in sepsis is substantially increased, and the more severe the AKI stage is, the higher the fatality rate is. AKI is an independent risk factor for the prognosis and increased risk of dying of severe sepsis. Therefore, strengthening the prevention and treatment of severe sepsis complicated with AKI is of great significance to improve the prognosis of patients.

At present, the diagnosis of severe sepsis complicated with AKI is mainly based on decreased urine volume and increased serum creatinine. Different countries and researchers have different definitions and diagnostic criteria for severe sepsis complicated with AKI, which brings some difficulties in the diagnosis, staging, and treatment of this disease [7–10]. Modern ultrasonic diagnosis technology has the advantages of being noninvasive, simple, and fast, having good repeatability, and allowing bedside examination. Abnormal changes in renal blood flow during AKI can indicate renal regulatory mechanisms. Studies showed that ultrasound diagnosis technology has high accuracy as an auxiliary method for the diagnosis of kidney diseases. Determination of the renal blood flow resistance index (RI) can reflect renal tubular necrosis in patients, which has a clinical application value for AKI diagnosis [11–13].

In recent years, with the continuous development of biological neuroscience, a new intelligent algorithm model, pulse-coupled neural network (PCNN), has emerged [14]. Due to the particularity of the biological background, spatial proximity, and similar brightness cluster, PCNN is very suitable for image processing. Combining the theoretical research results of PCNN with ultrasonic diagnosis technology is of great significance for the clinical diagnosis of severe sepsis complicated with AKI. The traditional noise filtering method destroys the detailed information of the image to a great extent, makes the edge of the image blurred, and reduces the quality of the target image to be processed. According to the characteristics of impulse noise, Cho et al. [15] proposed to combine mathematical morphology and peak-valley filtering into PCNN and apply them to ultrasonic image impulse noise processing, achieving a good denoising effect.

In this research, ultrasound diagnosis technology based on PCNN was innovatively applied to the image feature analysis of patients diagnosed with severe sepsis complicated with AKI. This research was aimed at improving the diagnostic accuracy and efficiency of severe sepsis complicated with AKI. It was hoped to investigate the clinical application value of the ultrasound diagnosis based on PCNN in patients with severe sepsis complicated with AKI.

## 2. Research Objects and Methods

### 2.1. Research Objects

In this research, 50 patients diagnosed with sepsis complicated with AKI in the hospital from May 2020 to June 2021 were collected as an observation group. There were 35 males and 15 females. The average age was 62.35 ± 12.14 years. Fifty patients with sepsis during the same period were selected as the control group, including 37 males and 13 females, aged 38-90 years, with an average age of 64.36 ± 13.46 years. This research had been approved by the ethics committee of the hospital. Patients and their families were aware of this study and have signed informed consent.

Inclusion criteria were as follows: (i) patients aged above 18, (ii) patients with clear consciousness and active cooperation, and (iii) patients with the course of disease less than 24 h.

Exclusion criteria were as follows: (i) those who had received renal replacement therapy before the experiment, (ii) pregnant or lactating women, (iii) those who used contrast media within five days before the experiment, (iv) patients requiring long-term hemodialysis treatment, and (v) patients with renal obstructive diseases and renal arterial organic diseases that affect renal blood flow.

### 2.2. Diagnostic Criteria

For severe sepsis, the diagnostic criteria were referred to in the *Guidelines for Emergency Treatment of Sepsis*/*Septic Shock in China* (2018) formulated by the Emergency Physicians Branch of the Chinese Medical Association and the Shock and Sepsis Professional Committee of the Chinese Society of Research Hospitals [16]: (i) body temperature over 38°C or below 36°C, (ii) heart rate over 90 beats/min, and (iii) respiration rate over 20 times/min or PaCO_2_ below 31.6 mmHg.

AKI was diagnosed based on the clinical guidelines developed by Kidney Disease: Improving Global Outcomes (KDIGO) [17]: (i) absolute value increase of sCr over 26 mmol/(L·48 h), (ii) increase of 1.5 times/week compared with the base value within 1 week, and (iii) urine volume below 0.5 mL/(kg·h) and over 6 h.

As for the diagnostic criteria for severe sepsis complicated with AKI, there is still no unified standard to distinguish severe sepsis complicated with AKI from nonseptic AKI, and it is generally accepted that both sepsis and AKI meet the above diagnostic criteria.

### 2.3. Observation Indexes

The clinical data of the two groups were collected, and the acute physiological and chronic health status assessment (APACHE II) score and sequential organ failure assessment (SOFA) score were compared between the two groups. APACHE II consists of the acute physiological score, age score, and chronic health score, with a score ranging from 0 to 71. The higher the score, the more severe the disease. The SOFA score uses six criteria to assess the respiratory, blood, liver, cardiovascular, nervous, and renal systems, which assigns each one a score of 0-4 on a scale of 6-24. The higher the score, the more severe the condition.

2 mL of fasting venous blood was taken from all confirmed patients the next day at 4,500 rpm, centrifuged for 20 min, and the supernatant was taken and stored in a refrigerator at -70°C. Serum creatinine, urea, and serum cystatin C levels were measured by a 7600 automatic biochemical analyzer (Hitachi Corporation, Japan).

### 2.4. Ultrasound Inspection Methods

All patients were examined by a color Doppler ultrasound diagnostic instrument on the first day of admission, with a probe frequency of 1-5 MHz. An ultrasonic contrast agent was used. Routine ultrasound examination was as follows. The patient was placed in the supine position, the kidney was fully exposed, and the scan measured the renal length diameter, renal transverse diameter, renal parenchymal thickness, and interlobular artery RI.

Contrast-enhanced ultrasound (CEUS) was used to observe the hilum and complete membrane and show a large area of the kidney. The long axial plane of the arcuate artery was selected to fix the ultrasonic probe. Then, local magnification was made, and it turned into real-time CEUS contrast pulse train mode. The contrast frequency was 1.5 MHz, the dynamic range was 85 dB, and the frame rate was 8 Hz. The superficial vein of the elbow on the opposite side of the kidney was selected, a 1.0 mL contrast agent was injected through the venous mass, and 5 mL normal saline was quickly and statically pushed. The timing was started when the contrast agent was injected, the dynamic images were observed and saved, and the development time was set at 2 min. The position of the ultrasonic probe was fixed, and the mean transit time (mTT) and perfusion index (PI) of the images were analyzed.

### 2.5. Ultrasound Based on the Artificial Intelligence Pulse-Coupled Neural Network Algorithm

In this research, the artificial intelligence-based PCNN algorithm was used to analyze the characteristics of ultrasonic image results. The PCNN neuron consists of three functional units of the feedback input domain, coupling connection domain, and pulse generator (Figure 1).

The input domain in the PCNN neuron model only receives input from the outside, and the expression of the input domain is as follows:

(1) $$\begin{array}{c} F_{ij}\left[m\right]=E_{ij}\left[m\right]. \end{array}$$

In equation (1), *F*_*ij*_[·] represents the feedback input of the *m*th iteration of the (*i*, *j*)th neuron, and *F* represents the transmission channel of *F*. *E*[·] represents the external input, *E* represents the *E* transmission channel, *ij* stands for the neuron, and the number of iterations is *m*.

Only pulse outputs of connected neurons are received in the connection domain of PCNN neurons, and the connection domain expression is as follows:

(2) $$\begin{array}{c} C_{ij}\left[m\right]=\underset{i}{\sum }W_{ij}Y_{i}\left[m\right]. \end{array}$$

In equation (2), *C*_*ij*_[·] represents the connection input of the *m*th iteration of the (*i*, *j*)th neuron, and *C* represents the *C* transmission channel. *W*_*ij*_ represents the weighting coefficient, *Y*_*i*_[·] represents the pulse output, and *Y* represents the *Y* transmission channel. *m* is the number of iterations.

The above two components simplify the receiving part of PCNN, which receives input from the outside and then transmits it through the transmission channel, respectively, so that the input of these two parts can be coupled in the modulation part.

### 2.6. Simulation Experiment and Image Segmentation Method

In this research, PCNN is introduced into the field of medical ultrasound image processing. According to the characteristics of ultrasound images, an ultrasound image enhancement algorithm based on PCNN is proposed by selecting appropriate parameters of PCNN to simulate the characteristics of human vision, and it is applied to the ultrasound image segmentation of patients with sepsis complicated with kidney injury [18].

To verify the effectiveness and practicability of the PCNN algorithm, this experiment used a large number of different types of images to perform computer simulation experiments on the MATLAB 7.0 platform. The experimental environment was a Win10 system, and the CPU was Intel® Celeron® CPU 1007U @ 1.50 GHz. The PCNN algorithm was compared with the results of the maximum between-class variance (OSTU) algorithm with better dynamic optimization capabilities and the maximum entropy algorithm with better segmentation results.

To quantitatively evaluate the processing results of different segmentation methods. This experiment took the following criteria to evaluate the effect of segmentation:

*(1) Regional Consistency (UM).* Quantitative analysis of segmentation results is performed, high-quality segmentation algorithms produce pixels within the segmentation area that should be consistent, and UM is calculated by calculating the feature variance within the area. The larger the value, the better the segmentation effect and the better the algorithm performance. UM is calculated as follows:

(3) $$\begin{array}{c} \text{UM}=1-\frac{1}{A}\overset{n}{\underset{i}{\sum }}{\left\lceil g\left(x,y\right)-\frac{1}{B}\overset{n}{\underset{i}{\sum }}g\left(x,y\right)\right\rceil }^{2}. \end{array}$$

In equation (3), *A* represents the normalization factor, *g*(*x*, *y*) represents the neighborhood grayscale function, *B* represents the normalization coefficient in the unit area, and *i* = 2 in the binary image.

*(2) Regional Contrast (CM)*. It can determine the difference between different regions in the segmentation result. The higher the value, the better the segmentation effect. CM is calculated as follows:

(4) $$\begin{array}{c} \text{CM}=\frac{\left|g_{a}-g_{b}\right|}{g_{a}+g_{b}}. \end{array}$$

In formula (4), *g*_*a*_ represents the average gray value of the target area and *g*_*b*_ represents the average gray value of the background area.

*(3) Region Shape Measure (SM).* The shape of the target region is evaluated by the edge, the edge of the target is extracted with different thresholds, and the segmentation effect is evaluated by observing the shape. The larger the value, the better the smoothness of the corresponding target contour and the better the segmentation effect. SM is calculated as follows:

(5) $$\begin{array}{c} \text{SM}=\frac{1}{A}\underset{\left(x,y\right)}{\sum }\mathrm{sgn}\left[g\left(x,y\right)-g_{L}\left(x,y\right)\right]\Delta \left(x,y\right)\mathrm{sgn}\left[g\left(x,y\right)-t\right]. \end{array}$$

In equation (5), *g*_*L*_(*x*, *y*) represents the mean gray value of the neighborhood *L*(*x*, *y*). *A* represents the normalization factor, Δ(*x*, *y*) represents the generalized gradient, and sgn(*x*) represents the sign function. *T* represents the gray threshold.

### 2.7. Statistical Methods

SPSS 19.0 was used for data processing. The measurement data conforming to normal distribution were expressed as mean ± standard deviation ($\overset{¯}{x}\pm s$), and the paired sample *t*-test was used between groups. The counting data were expressed in percentage (%), and the *χ*^2^ test was used to compare the difference between groups. *P* < 0.05 indicated that the difference was considerable.

## 3. Results

### 3.1. Simulation Experiment Results Based on the PCNN Algorithm

The OSTU algorithm is a global image enhancement algorithm, which can expand the grayscale of low-brightness ultrasound images and eventually produce excessive enhancement. The transformation function of the maximum entropy algorithm is simple, and the final image effect is not ideal. The proposed PCNN algorithm not only considers the global information but also enhances the local information. The gray value of the enhanced ultrasound image was evenly distributed around the sensitive gray value of human eyes, and the overall image effect was suitable for direct observation by naked eyes (Figure 2).

In terms of regional consistency (UM), regional contrast (CM), and shape measure (SM), the segmentation results of severe sepsis combined with AKI gray images using the PCNN algorithm were better than those of the OSTU algorithm and maximum entropy algorithm (*P* < 0.05, Figure 3).

### 3.2. General Statistics

Figure 4 shows the statistical results of general data. The observation group included 35 males and 15 females, with an average age of 62.35 ± 12.14 years. There were 37 males and 13 females in the control group, with an average age of 64.36 ± 13.46 years. There were no substantial differences in age and sex between the two groups (*P* > 0.05). The APACHE II score and SOFA score in the observation group were substantially higher than those in the control group, and the differences were great (*P* < 0.05). Among the 50 patients in the observation group, 29 cases (58%) were injured in road traffic accidents, followed by 11 cases (22%) of falling from high places, 2 cases (4%) of heavy objects, 6 cases (12%) of strangulation, and 2 cases (4%) of explosion.

### 3.3. Kidney Function Indexes

Figure 5 shows the comparison of renal function indexes between the two groups. 24 h urine volume in the observation group was substantially lower than that in the control group, and serum creatinine, urea, and serum cystatin C were substantially higher than those in the control group, and the differences were considerable (*P* < 0.05).

### 3.4. Analysis of CEUS Image Features

Figure 6 shows the CEUS images of patients with sepsis complicated with AKI. About 15 s after the contrast agent group injection, in the observation group of patients with sepsis complicated with AKI, it was observed that the trunk of the renal artery at the hilum began to enhance first, and the arteries of each layer in the kidney developed rapidly layer by layer, and finally, the cortex and medulla developed successively. The medulla was gradually enhanced from the periphery to the center, and the cortex was enhanced at the late stage of the medulla, showing rapid and uniform enhancement of the cortex. The medulla was the first to undergo contrast resolution, followed by the cortex.

### 3.5. Analysis of Related Indexes of Routine Ultrasound Examination

Figure 7 shows the comparative analysis of conventional ultrasound indexes. There were no substantial differences in the renal length diameter, renal transverse diameter, and renal parenchymal thickness between the observation group and the control group (*P* > 0.05), and the interlobular artery RI in the observation group was substantially higher than that in the control group (*P* < 0.05).

### 3.6. Quantitative Analysis of CEUS Indexes

Figure 8 shows the quantitative analysis of CEUS indexes. The mTT in the observation group was significantly higher than that in the control group (4.85 ± 1.27 vs. 3.42 ± 1.04), and the PI was significantly lower than that in the control group (134.46 ± 17.29 vs. 168.37 ± 19.28), with statistical significance (*P* < 0.05).

## 4. Discussion

AKI is the most common type of sudden renal impairment in patients with sepsis, which leads to the accumulation of toxins in the body and the dysfunction of multiple organs [19]. Serum creatinine, as one of the standard indexes reflecting kidney injury, has a good diagnostic value for patients with advanced kidney injury and has a certain predictive value for sepsis-related AKI [20–22]. Compared with serum creatinine, urine volume is a very sensitive index for evaluating kidney injury, which is more convenient for continuous monitoring and timely identification of kidney injury at an early stage. Atkinson [23] found that patients with a urinary volume less than 0.5 mL/(kg·h) sustained for 3-5 h could indicate the possibility of AKI. This study showed that the 24 h urine volume in the observation group was substantially lower than that in the control group, but the urine volume in both groups was in the normal range, indicating that the application of vasoactive drugs in patients had an impact on early fluid resuscitation. With improper infection control, the inflammatory response of sepsis patients gradually worsened, and the inflammatory factors released by the body further led to dilation of renal entering and leaving bulbous arterioles, hence leading to AKI. The degree of dilation of the bulbous arterioles is much greater, the degree of renal perfusion is reduced, and urine volume is constantly reduced, resulting in oliguria [24–26]. Serum cystatin C is a low-molecular weight protein secreted by eukaryotic cells that can pass freely through the glomerulus and be reabsorbed in the proximal renal tubules. Nishigawa et al. [27] found in their study that serum cystatin C can indicate AKI and was closely related to the glomerular filtration rate, which was one of the ideal markers reflecting the glomerular filtration rate.

In terms of regional consistency (UM), regional contrast (CM), and shape measure (SM), the segmentation results of the PCNN algorithm in this study were superior to the segmentation results of the OSTU algorithm and maximum entropy algorithm for severe sepsis combined with AKI gray images. Moreover, the PCNN algorithm not only considers the global information but also enhances the local information. The gray value of the enhanced ultrasound image was evenly distributed around the gray value sensitive to human eyes. The overall image effect was suitable for direct observation by naked eyes, which was consistent with the research results of Zhou et al. [28]. It indicated that the ideal image processing results can be obtained by using the artificial intelligence PCNN algorithm, which can provide clear ultrasound images for the clinical diagnosis, observation, and further analysis and processing of ultrasound images.

Conventional Doppler ultrasound is convenient and rapid to determine RI in patients with severe sepsis complicated with AKI. Therefore, renal perfusion is often assessed clinically by measuring RI at the interlobular artery level. It is generally believed that the normal value of renal RI is 0.60, and 0.70 is generally regarded as the upper limit of RI in normal adults. In this study, the renal RI score was measured for all enrolled patients. A convex array probe was used to obtain the right coronal section and transverse section of the kidney from a posterolateral abdominal scan to obtain the RI value. The results showed that according to KDIGO criteria for AKI diagnosis, the RI of the interlobular artery in the observation group was higher than that in the control group, and the difference was considerable (*P* < 0.05). This indicated that this method can be used to monitor renal perfusion in critically ill patients, which was similar to the results of Wang et al. [29].

CEUS is a new blood flow imaging method, which can timely detect and reflect the changes in the AKI renal blood perfusion state, and is more sensitive to small vascular lesions than conventional ultrasound. When AKI occurs in patients with severe sepsis, parameters related to contrast-enhanced renal ultrasound change. mTT refers to the time it takes for the ultrasound contrast agent to decrease from initial enhancement to half of the peak intensity of development. When early AKI occurs, the renal tubular epithelium appears edematous and the degree of necrosis increases, resulting in severe tubular obstruction in the lumen, contraction of the smooth muscle of the renal arterioles, and increased resistance to entering the bulbous arterioles. Finally, the contrast agent level in the renal cortex is lower than normal. The mTT of the observation group was substantially higher than that of the control group, the PI value was substantially lower than that of the control group, and the difference was considerable (*P* < 0.05). It indicated that in early AKI, the vascular perfusion of the renal cortex declines and PI decreases, while the stasis in the kidney leads to decreased metabolism of the contrast agent and increased mTT. Therefore, mTT and PI were sensitive in the diagnosis of AKI in sepsis patients.

## 5. Conclusion

Based on the ultrasonic image characteristics of the artificial intelligence PCNN algorithm, this paper compares and analyzes the inspection results. The PCNN algorithm can substantially increase ultrasonic image information. The RI value, mTT, and PI of the renal interlobular artery level in ultrasound images can be used as indexes for the diagnosis of severe sepsis complicated with AKI. However, the limitations of this study are that the sample size is small and it is a single-center study, so it needs to be expanded at a later stage to further promote the application of ultrasound in kidney injury. In conclusion, this study optimizes the ultrasound images of patients with severe sepsis complicated with AKI, providing a theoretical basis for future clinical trials and diagnosis.

## Figures and Tables

**Figure 1:** PCNN neuron model.

**Figure 2:** Ultrasound images of three algorithms: (a) OSTU algorithm, (b) maximum entropy algorithm, and (c) artificial intelligence PCNN algorithm.

**Figure 3:** Comparison of the three algorithms in measuring data. ^∗^Compared with PCNN, *P* < 0.05.

**Figure 4:** General statistics of the two groups of patients: (a) age and gender comparison, (b) APACHE II score comparison, and (c) SOFA score comparison. ^∗^Compared with the observation group, *P* < 0.05.

**Figure 5:** Comparison of renal function indexes between the two groups of patients: (a) 24 h urine output comparison, (b) serum creatinine comparison, (c) urea comparison, and (d) serum cystatin C comparison. ^∗^Compared with the observation group, *P* < 0.05.

**Figure 6:** CEUS images of patients with sepsis and AKI. (a) Patient 1, female, 56 years old. Acute tubular necrosis: cortical echo was enhanced, and kidneys were enlarged. (b) Patient 2, male, 58 years old. Acute renal trauma: laceration of the lower pole of the kidney, subcapsular effusion.

**Figure 7:** Comparative analysis of conventional ultrasound indexes. (a) Comparison of the renal long diameter, renal transverse diameter, and renal parenchymal thickness. (b) Comparison of interrenal artery RI. ^∗^Compared with the observation group, *P* < 0.05.

**Figure 8:** Quantitative analyses of CEUS indexes in the two groups: (a) mTT comparison and (b) PI comparison. ^∗^Compared with the observation group, *P* < 0.05.

## Data Availability

The data used to support the findings of this study are available from the corresponding author upon request.
